RETRACTED

# miR-141-3p Regulates EZH2 to Attenuate Porphyromonas gingivalis Lipopolysaccharide-Caused Inflammation and Inhibition of Osteogenic Differentiation in Human Periodontal Ligament Stem Cells

**DOI:** 10.1155/2022/4634925

**Published:** 2022-04-25

**Authors:** Zhu Zhu, Jie Xiong

**Affiliations:** Dongfeng Stomatological Hospital, Hubei University of Medicine, Shiyan, Hubei 442000, China

## Abstract

**Objective:**

miR-141-3p has been demonstrated to be both anti-inflammatory and osteoprotective. This study is aimed at investigating the effect of miR-141-3p on osteogenic differentiation of human periodontal ligament stem cells (hPDLSCs) stimulated by Porphyromonas gingivalis lipopolysaccharide (PgLPS) and its mechanism.

**Methods:**

PgLPS was used to induce an inflammatory environment, and overexpression of miR-141-3p was done to assess its effect on hPDLSCs in an inflammatory environment. The level of miR-141-3p and EZH2 in hPDLSCs from each treatment group was detected via qRT-PCR, and the inflammatory factors IL-6 and IL-8 in the supernatant of each group were detected by ELISA. ALP staining and alizarin red staining were used to assess the effect of miR-141-3p on the osteogenic differentiation ability of hPDLSCs, and also, western blot was used to detect expression of osteogenic differentiation-related proteins. Further, dual-luciferase reporter assay examined whether miR-141-3p targeted EZH2.

**Results:**

PgLPS led to a significant decrease of miR-141-3p in hPDLSCs. Overexpression of miR-141-3p could enhance ALP activity and alizarin red staining intensity and increase Runx2, OPN and OCN protein expression levels in PgLPS-treated hPDLSCs. Additionally, miR-141-3p could reduce IL-6 and IL-8. miR-141-3p could target and negatively regulate EZH2, and overexpression of EZH2 reversed the promoting effect of miR-141-3p on osteogenic differentiation.

**Conclusion:**

miR-141-3p can attenuate PgLPS-induced inhibition of osteogenic differentiation and inflammation in hPDLSCs by negatively regulating EZH2.

## 1. Introduction

Periodontitis is a chronic inflammatory disease caused by subgingival plaque accumulation and specific periodontal pathogens, which can progressively destroy the connective tissue around the teeth and cause stomatitis [1, 2]. If the initial inflammatory response is not adequately resolved, periodontitis will cause destruction of alveolar bone, periodontal ligaments, and cementum, ultimately leading to tooth loss [3, 4]. According to epidemiological surveys, periodontitis is currently one of the six most common diseases in the world, affecting about 734 million people with an overall prevalence of 11.2%, and the global prevalence of periodontal diseases has been growing rapidly in the past two decades [5, 6].

RETRACTED

Periodontal ligament stem cells (PDLSCs) are a class of heterogeneous pluripotent stem cells with physiological self-replication capacity and multilineage differentiation potential [7]. PDLSCs can potentially differentiate into multiple cell types, especially osteoblasts or cementoblasts. Studies have shown that PDLSC can be applied to periodontal regeneration in dogs, rats, and sheep [7]. Sano et al. found that cocultured PDLSCs with umbilical vein endothelial cells revealed that cocultured spheroids enhanced periodontal tissue regeneration [8]. Some experimental evidence has also confirmed that osteogenic differentiation of PDLSCs can improve periodontal tissue regeneration, providing important application value for bone tissue maintenance, bone regeneration, and periodontal tissue repair in dental clinical practice [9–11].

MicroRNAs (miRNAs), a class of conserved endogenous noncoding small RNAs of about 21–25 nt in length, are found in eukaryotes and can regulate gene expression by posttranscriptional control [12]. miRNAs are involved in regulating various physiological and pathological processes such as cell proliferation, differentiation, apoptosis, inflammation, tumorigenesis, and tumor progression [13]. According to researches, a variety of miRNAs are involved in regulating the homeostasis and pathological processes of periodontal tissue and play a coordinating role in periodontal tissue inflammation and bone remodeling through different pathways [14, 15].

miR-141-3p was demonstrated to lower expression in the gingiva of periodontitis patients [16]. However, its expression, function, and molecular regulatory mechanism during osteogenic differentiation of hPDLSCs are unknown. Therefore, in this study, the regulatory function of miR-141-3p on osteogenic differentiation of hPDLSCs in an inflammatory environment was explored with PgLPS-induced hPDLSCs as a model of periodontitis. Our study provides an important theoretical basis for explaining the osteogenic differentiation of hPDLSCs under inflammatory conditions and how to promote oral tissue regeneration. Also, our results contribute to the development of new ideas and treatments of using hPDLSCs for tissue regeneration.

## 2. Methods

### 2.1. Cell Culture

hPDLSCs were obtained from the American Type Culture Collection (ATCC) and cultured in ɑ-MEM medium (Gibco, USA) containing 10% fetal bovine serum (FBS; Gibco, USA) at 37°C in a 5% CO_2_ incubator. The cell culture medium was changed every 3 days.

### 2.2. Cell Transfection

miR-141-3p mimic and its negative control (100 nM), miR-141-3p inhibitor and its negative control (100 nM), and pcDNA3.2-EZH2 and no-load pcDNA3.2 (2 *μ*g) were purchased from GenePharma (Shanghai, China). Cells with 70%-80% confluence in 6-well plates were transfected according to the instructions of Lipofectamine 2000 reagent (Invitrogen, Carlsbad, CA, USA). Cells were divided into 6 groups, and PgLPS treatment was carried out 24 h after transfection [1]: control group: no PgLPS, no transfection [2]; PgLPS group: 1 *μ*g/ml PgLPS, no transfection [3]; PgLPS+NC mimic group: 1 *μ*g/ml PgLPS, cells transfected with negative mimics [4]; PgLPS+miR-141-3p mimic group: 1 *μ*g/ml PgLPS, cells transfected with miR-141-3p mimics [5]; PgLPS+miR-141-3p+pcNC group: 1 *μ*g/ml PgLPS, cells transfected with miR-141-3p mimics and negative pcDNA3.2 [6]; and PgLPS+miR-141-3p+EZH2 group: 1 *μ*g/ml PgLPS, cells transfected with miR-141-3p mimics and pcDNA3.2-EZH2.

RETRACTED

### 2.3. ELISA

Cell culture supernatants were collected from each group, and cell debris removed by centrifugation. The levels of IL-6 and IL-8 in the supernatant were measured with ELISA kits (Multisciences Biotech), and all operations were performed in strict accordance with the instructions.

### 2.4. qRT-PCR

Cells and tissue samples were collected, and total RNA was extracted by using TRIzol (Invitrogen, Carlsbad, CA, USA). Reverse transcription was performed by using a reverse transcription kit (TaKaRa, Tokyo, Japan), and all operations were performed according to the instruction. The expression of target genes was detected with LightCycler 480 qRT-PCR (Roche, Indianapolis, IN, USA), and reaction conditions were performed according to the instructions of the qRT-PCR kit (SYBR Green Mix, Roche Diagnostics, Indianapolis, IN). Thermal cycling parameters were as follows: 95°C for 10s, 45 cycles of 95°C for 5 s, 60°C for 10s, 72°C for 10 s, and 72°C for 5 min. Three replicates per reaction were set up for qRT-PCR. GAPDH was used for internal reference. Data analysis was performed by the 2^-*ΔΔ*Ct^ method, where ΔΔCt = treatment group (Ct target gene − Ct internal reference)–control group (Ct target gene − Ct internal reference). The sequences of the amplimers for each gene and the internal reference are listed in Table 1.

### 2.5. Osteogenic Induction

Third-passage hPDLSCs were evenly seeded in 24-well culture plates, and when confluence reached 60%-70%, the cell culture medium was replaced with osteogenic induction solution to induce cell differentiation into osteoblasts. The solution was changed every 2-3 two days; the induction was carried out for 1, 3, 7, 14, and 24 days, respectively. Alkaline phosphatase staining (on day 7 of induction) and alizarin red staining (on day 21 of induction) were then completed. The formulation of osteogenic induction solution was as follows: adding vitamin C (100 *μ*M), P-sodium glycerophosphate (10 mM), and dexamethasone (10 nM) into *α*-MEM complete medium containing 10% FBS.

RETRACTED

### 2.6. Alkaline Phosphatase (ALP) Staining and Activity Detection

First, PBS was used to rinse hPDLSCs on day 7 of osteogenic differentiation and then aspirated. Then, fixing solution was added and incubated with the cells for 30 min. Next, ALP staining solution was added to the plates for incubation at room temperature for 12 min, and the incubation was protected from light. On completion of incubation, the cells were rinsed with ddH_2_O, and counterstaining was performed if necessary. After successful staining, the cells were dried to observe the staining of cells. The activity of ALP was detected with ALP activity kit (Beyotime, Shanghai, China) according to the manufacturer's protocol.

### 2.7. Alizarin Red Staining

First, PBS was used to rinse hPDLSCs on day 7 of osteogenic differentiation and then aspirated. Then, 4% paraformaldehyde was added and incubated with the cells for 30 min. After rinsing step with ddH_2_O, 2% alizarin red staining solution with a pH of 4.24 was then added into the cell culture plate for 8-15 min staining at room temperature. Next, the staining solution was aspirated, followed by rinsing step using ddH_2_O; counterstaining was performed if necessary. The cells were dried to observe the formation of the mineralized nodule and quantified calcium level with spectrophotometry at 562 nm.

### 2.8. Western Blot

Cells were lysed with RIPA lysis solution (Beyotime) to obtain protein samples. After measuring protein concentration with BCA kit (Beyotime), the protein was added into a corresponding volume of loading buffer (Beyotime) and fully mixed. The mixture was heated in boiling water for 5 min to denature proteins. Then, proteins were transferred to PVDF membrane, followed by 1 h blocking using 5% nonfat dry milk. Primary antibodies (GAPDH (5174S, 1 : 1000, Cell Signaling, Boston, USA), RUNX2 (# 12556S, 1 : 1000, Cell Signaling, Boston, USA), OPN (ab8448, 1 : 1000, Abcam, Boston, USA), OCN (ab133612, 1 : 1000, Abcam, Boston, USA), and EZH2 (# 5246S, 1 : 1000, Cell Signaling, Boston, USA)) were added into the membrane and incubated overnight at 4°C. The next day, the membrane was rinsed 3 times prior to 1 h incubation with secondary antibodies (horseradish peroxidase-labeled IgG, 1 : 5000, Beijing CoWin Biosciences Co., Ltd., China, Beijing) at room temperature. After the developer was dropped on the membrane, the detection was performed by chemiluminescence imaging system (Bio-Rad).

### 2.9. Dual-Luciferase Reporter Assay

Through the online database TargetScan (http://www.targetscan.org/vert_72/), the binding site of miR-141-3p and EZH2 was predicted. According to the predicted results, the wild sequence and mutant sequence (mut-EZH2, wt-EZH2) of the binding site were designed and synthesized, respectively. These sequences were inserted into the luciferase reporter gene vector (pGL3-Basic), respectively, and then cotransfected HEK293T cells with miR-141-3p mimic (0, 150 nM, 300 nM, GenePharma), respectively. After mixing well, 100 *μ*l of cell lysis solution was added and the cells were allowed to fully lyse on a shaker for 20 min at room temperature. 50 *μ*l of luciferase reaction solution (Promega, Madison WI, USA) was added to 50 *μ*l of lysed cells to measure Firefly luciferase activity, while 50 *μ*l of Stop & Glo reagent (Promega, USA) for detecting Renilla luciferase activity. Renilla luciferase activity was used as an internal reference, and the ratio of Firefly luciferase activity to Renilla luciferase activity was the relative activity of luciferase. Three replicates were set up for the experiment.

RETRACTED

### 2.10. Statistical Analysis

The experimental data were shown in the form of mean ± standard deviation (SD). One-way analysis of variance (one-way ANOVA) was performed by using GraphPad Prism 8.0 software, and multiple comparisons of the mean were carried out with the Tukey method. The result difference was considered to have statistical significance if *P* < 0.05.

## 3. Results

### 3.1. Isolation and Identification of Human Periodontal Ligament Stem Cells (hPDLSCs)

Primary cells were scattered somewhere at the bottom of the culture flask or around tissue blocks (Figure 1(a)). Most of the cells were cord-like, long, and spindle-like in shape, with plump cell body, round or oval nuclei, and distinct and visible nucleoli. After about 5-10 days of culture, the adherent cells swirled and grew radially around tissue blocks, with a rapid growth rate. Even some cells fused with each other and showed multilayer growth, and at this time, the ratio of 1 : 1 could be selected for subculture. The flow cytometry showed the positive expression of hPDLSC surface antigens CD73 and CD90 and negative expression of CD45, suggesting that hPDLSCs were successfully isolated (Figures 1(b)–1(c)).

### 3.2. miR-141-3p Attenuates PgLPS-Caused Inhibition of Osteogenic Differentiation in hPDLSCs

The expression of miR-141-3p in each treatment group was detected by qRT-PCR. The results showed that miR-141-3p was significantly downregulated in hPDLSCs treated with PgLPS, while it increased significantly after transfection of miR-141-3p mimics (Figure 2(a)). The results of ALP and alizarin red staining showed that PgLPS treatment significantly inhibited the osteogenic differentiation ability of hPDLSCs, and the inhibitory effect was alleviated after miR-141-3p overexpression (Figures 2(b)–2(e)). Then, the protein levels of osteogenic markers were detected with western blot. Protein expression levels of Runx2, OPN, and OCN were significantly decreased after PgLPS treatment, while they increased after miR-141-3p overexpression (Figures 2(f) and 2(g)).

RETRACTED

### 3.3. miR-141-3p Attenuates Inflammation Induced by PgLPS

After PgLPS treatment, the levels of IL-6 and IL-8 were significantly increased. Compared with the PgLPS+NC mimic group, their expression showed a marked reduction in the PgLPS+miR-141-3p mimic group, indicating that miR-141-3p could attenuate the inflammatory response induced by PgLPS (Figures 3(a) and 3(b)).

### 3.4. miR-141-3p Targets EZH2

The levels of EZH2 in the cells of each treatment group were measured by qRT-PCR (Figure 4(a)). PgLPS treatment significantly increased EZH2 level while transfection of miR-141-3p caused a decrease of its expression level.  Figure 4(b) showed the targeted binding site of miR-141-3p and EZH2, and dual-luciferase reporter assay further validated that miR-141-3p targeted EZH2 (Figure 4(c)).

### 3.5. EZH2 Reverses the Therapeutic Effect of miR-141-3p on PgLPS-Induced hPDLSCs

The results of ALP and alizarin red staining showed that miR-141-3p overexpression increased the osteogenic activity of hPDLSCs, and EZH2 counteracted this promoting effect (Figures 5(a)–5(d)). The effect of EZH2 on the inflammatory response of hPDLSCs was confirmed by using ELISA analysis. The results showed that compared with the PgLPS group, the levels of IL-6 and IL-8 in the PgLPS+miR-141-3p+pcNC group were significantly decreased; compared with the PgLPS+miR-141-3p+pcNC group, their expression was significantly increased in the PgLPS+miR-141-3p+EZH2 group (Figures 5(e) and 5(f)). The result of western blot indicated that the promoting effect of miR-141-3p on Runx2, OPN, and OCN protein expression could be reversed by upregulating EZH2 (Figures 5(g) and 5(h)).

## 4. Discussion

Periodontitis is a destructive periodontal inflammatory disease characterized pathologically by periodontal tissue inflammation, periodontal pocket formation, alveolar bone resorption, and progressive attachment loss [17] Plaques contribute to the development of periodontitis, but plaques not fully account for this development. Sufficient evidence has shown that the occurrence of periodontitis is an excessive inflammatory response (immune response) of the host to pathogenic microorganisms and their toxic products, further leading to periodontal tissue destruction. Once periodontal tissues are lost, the primary goal of periodontal therapy is to regenerate diseased tissues into their original form, structure, and function as far as possible [18].

RETRACTED

PDLSCs are a kind of undifferentiated mesenchymal stem cells in the periodontal ligament with the potential to differentiate into osteoblasts or cementoblasts. PDLSCs can form cementum-periodontium-alveolar bone-like structures *in vivo*, thus constructing new periodontal tissue structures and rebuilding periodontal attachment [9, 19]. Therefore, PDLSCs become ideal candidates for cell therapy for treating injuries due to trauma or periodontal diseases [20]. The occurrences of many inflammatory diseases and autoimmune diseases are associated with defects in mesenchymal stem cell function *in vivo* [21]. Lipopolysaccharide induces the expression of proinflammatory cytokines during inflammation, which in turn promotes apoptosis to reduce the proliferation rate of mesenchymal stem cells [22]. PDLSCs interact with the inflammatory microenvironment to regulate cell stemness, proliferation, migration, differentiation, immunoregulatory attributes, and the Wnt pathway, and the interaction and subsequent regulation may be a potential cause affecting periodontal tissue regeneration and repair [23]. A study shows that the inflammatory environment induced by PgLPS can promote the secretion of TNF-*α*, IL-8, and IL-18 from hPDLSCs [24], which is consistent with our findings. In addition, our study demonstrated that PgLPS induction significantly inhibited the osteogenic activity of hPDLSCs and decreased the protein levels of osteogenic markers.

An increasing body of evidence has suggested that miRNAs can regulate the differentiation potential of stem cells through posttranscriptional mechanisms [25]. At present, miRNAs have been found to be involved in the regulation of osteogenic differentiation and bone formation in a variety of cells [26, 27]. Li et al. demonstrated that miR-141-3p is important for osteogenic differentiation of stem cells from the apical papillae (SCAPs) [28]; miR-141-3p inhibits the proliferation of SCAPs and accelerates cellular senescence by downregulating the expression of YAP [28]. Recently, it has been found that knockdown of miR-141-3p can promote the proliferation level of mesenchymal stem cells by upregulating the expression of *β*-catenin, C-Myc, and cyclin D1 [29]. Despite these findings, the effect of miR-141-3p on the osteogenic differentiation ability of hPDLSCs under an inflammatory microenvironment has not been elucidated. Our current study found that miR-141-3p was significantly downregulated in hPDLSCs treated with PgLPS; miR-141-3p overexpression significantly increased the osteogenic differentiation activity of hPDLSCs treated with PgLPS and inhibited the secretion of proinflammatory cytokines IL-6 and IL-8. Additionally, Runx2, OPN, and OCN osteogenic marker proteins were significantly increased in hPDLSCs with the overexpression of miR-141-3p, also demonstrating the stimulatory effect of miR-141-3p on osteogenic activity of hPDLSCs in periodontitis.

miRNAs can exert biological functions by regulating downstream target genes. EZH2 or enhancer of zeste homolog 2 is a histone methyltransferase that plays an important role in maintaining the self-renewal and proliferation ability of stem cells [30]. EZH2 has been validated to promote the migration of bone marrow stem cells by increasing the level of H3 lysine 27 trimethylation (H3K27me3) [31]. Ma et al. believed that EZH2 overexpression enhances migration and chemotaxis of SCAPs and that SCAPs enhance homing, migration, and chemotaxis of hPDLSCs through paracrine signaling [32]. Upregulation of EZH2 induced by lipopolysaccharide inhibits osteogenic activity of hPDLSCs under inflammatory conditions through the Wnt/*β*-catenin pathway [33]. By contrast, inhibition of EZH2 not only promotes osteogenic differentiation of progenitor cells mediated by BMP2 but also enhances osteogenesis and myogenic regeneration by regulating the expression of differentiation genes [34, 35]. In this study, the dual-luciferase reporter gene assay proved that EZH2 was a downstream target of miR-141-3p, and it found that overexpression of EZH2 reversed the stimulatory effect of miR-141-3p on osteogenic differentiation of hPDLSCs under an inflammatory microenvironment.

RETRACTED

In conclusion, miR-141-3p can attenuate PgLPS-induced inhibition of osteogenic differentiation and inhibit secretion of IL-6 and IL-8 in hPDLSCs. These effects of miR-141-3p are achieved by negatively regulating EZH2. Therefore, the miR-141-3p/EZH2 axis can be a potential target for the treatment of periodontitis.

## Figures and Tables

**Figure 1:** Isolation and identification of hPDLSCs. (a) hPDLSCs isolated from periodontal ligament tissue; (b, c) Flow cytometry-based detection of hPDLSC markers CD45, CD37, and CD90.

**Figure 2:** miR-141-3p attenuates PgLPS-caused inhibition of osteogenic differentiation in hPDLSCs. (a) qRT-PCR-based measurement of miR-141-3p expression; (b, d) ALP staining and ALP activity levels; (c, e) alizarin red staining and quantification of calcium level; (f, g) western blot-based detection of Runx2, OPN, and OCN protein expression. ^∗^*P* < 0.05 and ^∗∗^*P* < 0.01.

**Figure 3:** miR-141-3p attenuates the inflammatory response induced by PgLPS. (a, b) ELISA assay for IL-6 (a) and IL-8 (b) expression. ^∗^*P* < 0.05 and ^∗∗^*P* < 0.01.

RETRACTED

**Figure 4:** miR-141-3p targets EZH2. (a) qRT-PCR-based measurement of mRNA levels of EZH2 in the cells of each group. (b) The predicted binding site of miR-141-3p and EZH2. (c) Dual-luciferase reporter gene assay was performed after hPDLSCs were cotransfected with luciferase reporter genes containing mut-/wt-EZH2 and miR-141-3p mimics. ^∗^*P* < 0.05 and ^∗∗^*P* < 0.01.

**Figure 5:** EZH2 reverses the therapeutic effect of miR-141-3p on PgLPS-induced PDLSCs. (a, b) ALP staining and ALP activity levels of cells in each group; (c, d) alizarin red staining and quantification of calcium level; (e, f) ELISA assay for IL-6 and IL-8 expression; (g, h) western blot detection of Runx2, OPN, and OCN protein expression. ^∗^*P* < 0.05 and ^∗∗^*P* < 0.01.

**Table 1:** Primer sequences.

Primer		Sequence (5′-3′)
miR-141-3p	Forward	CTTCCAGTACAGTGTTGG
	Reverse	GAACATGTCTGCGTATCTC
U6	Forward	UUCUCCGAACGUGUCACGUTT
	Reverse	UGACACGUUCGGAGAATT
EZH2	Forward	GACCTCTGTCTTACTTGTGGAGC
	Reverse	CGTCAGATGGTGCCAGCAATAG
GAPDH	Forward	GGAGCGAGATCCCTCCAAAAT
	Reverse	GGCTGTTGTCATACTTCTCATGG

## Data Availability

The data used to support the findings of this study are available from the corresponding author upon request.
